The article "The Supervision and Management Mode of Disinfection Supply Center Improves the Standardization of Sterile Goods Management in Clinical Departments" was retracted in 2023. Reasons: unreliable results or conclusions; concerns about the data; concerns about the results or conclusions; concerns about the peer review.

# The Supervision and Management Mode of Disinfection Supply Center Improves the Standardization of Sterile Goods Management in Clinical Departments

**DOI:** 10.1155/2022/6916212

**Published:** 2022-02-15

**Authors:** Jia Ying, Haiying Wang, Hui Ye, Cuiqi Du, Lili Mao

**Affiliations:** Department of Central Sterile Supply, Affiliated Hangzhou First People's Hospital, Zhejiang University School of Medicine, 310006 Hangzhou, China

## Abstract

**Background:**

In daily inspection, the nonstandard management of sterile articles in clinical departments of hospitals often leads to the destruction of the sterilization effectiveness of sterile articles. Therefore, it is necessary to strengthen governance and improve this phenomenon. This study intends to investigate the mode in which the disinfection supply center participates in the supervision and management of the management of sterile items in clinical departments. It played a role in improving the standardization of the management of sterile articles in clinical departments and ensured the closed-loop management of the sterilization effectiveness of sterile articles.

**Methods:**

Every quarter, the disinfection supply center of our hospital will inspect the standardized management of sterile articles in all clinical departments of the hospital, mainly including the storage environment and facilities of sterile articles, the cleanliness of storage cabinets, placement principles, whether they are stored by category, and the quality and validity management of sterile articles. The quarterly inspection results were summarized and analyzed to find the existing problems and the causes. The disinfection supply center shall supervise the improvement. After the disinfection supply center inspected the standardized management of sterile articles in all clinical departments of the hospital for the first time according to the inspection contents, under the guidance and assistance of the nursing department and the hospital infection department, it improved the sterile article management system, conducted knowledge training for the whole hospital, and incorporated the standardized management of clinical sterile articles into the quality control inspection of the nursing department. In the later stage, the disinfection supply center is responsible for conducting routine inspection and supervision on the standardized management of sterile articles in all clinical departments of the hospital every quarter according to the inspection contents, including summarizing, analyzing, and urging the clinical departments to achieve the improvement of the management of sterile articles in clinical departments.

**Results:**

The standardization of aseptic articles after improvement was significantly higher than before and during improvement, and the qualified rate was significantly different (99.4% vs 97.9% vs 89.5%, *P* < 0.05). The average number of lost packages caused by nonstandard management in the department was significantly reduced. The average rate of lost sterile packages during and after the improvement was significantly lower than that before the improvement (10.5% vs 97.9% vs 89.5%, *P* < 0.05). It also effectively reduced the cost caused by the loss of sterile packages.

The article "The Supervision and Management Mode of Disinfection Supply Center Improves the Standardization of Sterile Goods Management in Clinical Departments" was retracted in 2023. Reasons: unreliable results or conclusions; concerns about the data; concerns about the results or conclusions; concerns about the peer review.

**Conclusion:**

The disinfection supply center participates in the quality control and management of sterile articles in the nursing department and regularly inspects and supervises the management of sterile articles in clinical departments. It can effectively improve the standardized management of sterile articles in clinical departments, ensure the safety of sterile articles, and form a closed loop of sterilization effectiveness.

## 1. Introduction

The disinfection supply center is one of the key departments of the hospital, an important department in nosocomial infection management [1] and an essential part of hospital cost accounting. The storage of sterile articles is also a critical work content of the disinfection supply center [2] and has rich theoretical knowledge and practical experience in sterile article management [3]. Objects in contact with damaged skin, mucous membrane, tissue, and organ through the skin or mucous membrane shall be sterilized [4]. The objects after sterilization are called sterile articles. Generally, the disinfection supply center develops a traceability system for sanitary articles. The relevant records of the quality control process should be improved to ensure the safety of articles [4]. With the development of hospital informatization, the informatization traceability system is basically used for the quality control process of sterile articles. The system records the whole closed-loop management of article recovery, cleaning, packaging, sterilization, storage, distribution, and use, which can effectively standardize the workflow of the disinfection supply center and clinical departments. The system can comprehensively improve the quality of sterile articles [5]. However, the clinical departments lack quality supervision on managing sterile articles before use. During the inspection, we found many aspects that need improvement. To ensure the effective and safe use of sterile articles, we adopted the supervision and management mode of disinfection supply center for the first time to supervise and inspect the management of sterile articles in clinical departments. The disinfection supply center analyzed the causes of the deficiencies found in the inspection according to the professional knowledge, improved the sterile goods management system under the guidance of the nursing department and the hospital feeling department, conducted knowledge training, and carried out routine quarterly inspection and guidance improvement on the sterile goods in the clinical departments. The results are promising. It is reported as follows.

The article "The Supervision and Management Mode of Disinfection Supply Center Improves the Standardization of Sterile Goods Management in Clinical Departments" was retracted in 2023. Reasons: unreliable results or conclusions; concerns about the data; concerns about the results or conclusions; concerns about the peer review.

## 2. Materials and Methods

### 2.1. General Information

The Affiliated Hangzhou First People's Hospital, Zhejiang University School of Medicine is a class III class a comprehensive hospital. 65 clinical departments use the sterilized articles of the disinfection supply center. Three senior nurses of the disinfection supply center conduct special inspections on the management of sterile articles in these departments, mainly routine standby sterile bags, special bags, and special sterile articles for emergency rescue, which are uniformly placed in the cabinet of the treatment room.

## 3. Methods

### 3.1. Identify Problems and Analyze Causes

According to the specifications for disinfection supply center and the on-the-job training course for hospital disinfection supply center, the inspection contents mainly include the following: (1) According to the expiration date, place them in an orderly manner from left to right, follow the principle of first-in, first-out, and take out the expired package in time. (2) The storage environment requires the temperature to be lower than 24°C and the humidity to be lower than 70%, sterile items are stored, the height from the ground is required to be ≥20 cm, the distance from the wall is ≥5 cm, and the distance from the ceiling is ≥50 cm. (3) Sterile items should be classified and stored in separate cabinets, and the storage cabinets should be kept clean and dry. (4) According to the needs of the department and the cost, determine the sterility of each department pack base and record. (5) The department is required to count the number of sterile packs every day and check the quality. If the outer packaging is loose and damaged, and the label is incomplete, take it out in time. From April to June 2018, the staff of the disinfection supply center inspected 65 clinical departments. The inspection mainly adopts the method of on-site assessment and hearing from the staff of the Inquiry Department. The inspection results are summarized and analyzed by the disinfection supply center and the nursing department. The main problems are shown in Table 1. The nursing department and the disinfection supply center analyzed the leading causes of the problems: (1) Many department managers and users ignored the importance of the base number of sterile bags. (2) The clinical staff lacked knowledge about the storage and use of sterile articles and expired bags stored in the sterile bags. (3) The cabinets where the sterile bags were placed did not remove dust in time, and some are very old. (4) The distribution in the disinfection supply center and the counting in the department are not standardized, resulting in loose packaging of sterile bags, damaged labels, and even possible damage of sterile bags. (5) The nursing department does not have specialized personnel to inspect sterile articles, and the department managers lack adequate supervision on this work.

The article "The Supervision and Management Mode of Disinfection Supply Center Improves the Standardization of Sterile Goods Management in Clinical Departments" was retracted in 2023. Reasons: unreliable results or conclusions; concerns about the data; concerns about the results or conclusions; concerns about the peer review.

### 3.2. Take Corresponding Measures for Improvement

The nursing department incorporated the standardized management of clinical, sterile articles into the quality control inspection of the nursing department. The disinfection supply center is responsible for conducting routine inspection and supervising improvement according to the inspection contents every quarter. It was analyzed and discussed at each quality control meeting of the nursing department. Some departments carried out continuous quality improvement for the standardized management of sterile articles to urge the department managers to strengthen the standardized supervision of sterile articles.

The head nurse of the disinfection and supply center gave standardized teaching and on-site training on the management of sterile articles to the head nurses of clinical departments and senior nurses of the whole hospital. They introduced the standardized operation of the management of sterile articles in the disinfection and supply center and the identification of sterilization effectiveness. Then, let the trainees return to the department for secondary training and popularize it to every staff member. The teaching and training contents mainly include the importance of storage and use of sterile articles, the necessity of overall arrangement of the base package, storage environment, facility requirements, placement and taking requirements, influencing factors, and other related knowledge. The relevant training contents were included in the theoretical examination of the nursing department to evaluate the learning effect of nursing staff. This measure enables the clinical department personnel to understand and improve the standardized management of sterile articles in theory and practice.

The process started with the staff of the disinfection supply center, which set an example and strictly controlled sterile articles' quality. They ensured that the indication tape outside the sterilization package could be distributed to the clinical department only after it was discoloured and qualified. The process required the special frame to be sealed for transportation, strictly implemented hand hygiene when taking it, paid attention to the clean and dry placement position, and handled it gently to avoid damaging the packaging of the sterile package. In case of any problem, communicate with the clinical department in time and put forward any nonstandard operation. At the same time, the sterilization indication discoloration comparison card made by the disinfection supply center was distributed to the clinical department so that the clinical department staff could know the discoloration requirements of the indication card inside and outside the sterile package and make a good judgment.

The article "The Supervision and Management Mode of Disinfection Supply Center Improves the Standardization of Sterile Goods Management in Clinical Departments" was retracted in 2023. Reasons: unreliable results or conclusions; concerns about the data; concerns about the results or conclusions; concerns about the peer review.

The disinfection supply center can improve the existing sterile article management system and refine the distribution and receiving process, and the hospital infection control department will assist in the audit. Finally, the nursing department can distribute the sterile article management system to all clinical departments for homogenization and implementation.

During the rectification process, for the more prominent problems in each inspection, such as the inconsistency between the base number of sterile bags and the records, the on-site rectification shall be carried out immediately, and the importance of fixing the base number of sterile bags shall be emphasized again during the lecture. The actual number shall be consistent with the base number. If the base number is insufficient, the disinfection supply center shall be informed to increase it in time to facilitate overall arrangement and save hospital costs.

### 3.3. Inspection during Improvement

During the year from July 2018 to June 2019, after the implementation of the measures, the disinfection supply center conducted routine supervision, summary and rectification on the management of sterile articles in the clinical departments of the whole hospital every quarter, four times in total, and timely put forward the nonstandard management of sterile articles in the clinical departments during the normal distribution process. According to the actual situation in the implementation of the inspection, the focus of the inspection content was appropriately adjusted, the inspection of the damage of the sterile package was strengthened, and the results of the four inspections under improvement were summarized so as to evaluate the feasibility of the supervision model of the disinfection supply center.

### 3.4. Inspection after Improvement

After determining the feasibility of the supervision model of the disinfection supply center in the standardized management of sterile articles in clinical departments, with the assistance of the nursing department and the hospital feeling department, the disinfection supply center will continue to inspect the standardized management of sterile articles in clinical departments of the whole hospital every quarter, supervise and correct problems, and summarize and score at the same time. The special management of sterile articles was included in the quality control inspection of the nursing department. By summarizing the results of 8 inspections from July 2019 to June 2021, we can further evaluate the effect and significance of the supervision model of the disinfection supply center in the standardized management of sterile articles in clinical departments.

The article "The Supervision and Management Mode of Disinfection Supply Center Improves the Standardization of Sterile Goods Management in Clinical Departments" was retracted in 2023. Reasons: unreliable results or conclusions; concerns about the data; concerns about the results or conclusions; concerns about the peer review.

### 3.5. Summary of Inspection Content

Composition ratio = frequency of problems/total frequency of problems × 100%. Qualified rate of inspection results = total qualified frequency/total inspection frequency × 10%. Loss package rate = average number of lost packages/total number of single inspection packages × 100%. The loss value is the single loss value = the average number of lost packages × unit price.

### 3.6. Statistical Analysis

SPSS22.0 was used for statistical analysis. The counting data were expressed in percentage and compared between groups *χ*^2^ test, *P* < 0.05; the difference was statistically significant.

## 4. Results

Three training sessions were conducted for the clinical departments of the hospital. The number of participants and clinical departments are shown in Table 2.

During the rectification process from July 2018 to June 2019, the disinfection supply center was responsible for the statistics of the results of four rounds of quarterly inspection on the standardized management of sterile articles in 65 clinical departments of the hospital. The existing problems were less than those before the rectification, as shown in Table 3.

From July 2019 to September 2021, after rectification, the disinfection supply center was responsible for 8 rounds of standardized management of sterile articles in 65 clinical departments, and the quarterly inspection results were counted. The existing problems were less than those before and during the rectification, as shown in Table 4.

The results of the standardized inspection of sterile articles in each clinical department were summarized and compared the qualification rates of the three processes, as shown in Table 5. Before, during, and after rectification are 89.5% vs 97.5% vs 99.4%, respectively. Compare the number (rate) of sterile packages lost by the clinical department due to nonstandard management in the three processes, before, during, and after rectification is 10.5% vs 97.9% vs 89.5% and corresponding values, respectively, see Table 6*P* < 0.05 in *χ*^2^ test, indicating the difference is statistically significant.

The article "The Supervision and Management Mode of Disinfection Supply Center Improves the Standardization of Sterile Goods Management in Clinical Departments" was retracted in 2023. Reasons: unreliable results or conclusions; concerns about the data; concerns about the results or conclusions; concerns about the peer review.

## 5. Discussion

With the development of medical technology, the disinfection supply center has become an essential department for the hospital's development and a guarantee for sterile articles in the hospital. It provides cleaning, disinfection, sterilization, and disposable sterile articles for all hospital departments [6–8]. Therefore, the disinfection supply center has strong professionalism in the standardized management of sterile articles and fully understands the significance of the standardized management of sterile articles. At the same time, the disinfection supply center should strictly control the standardization of the whole process of the use of sterile articles [9, 10]. Studies have shown that the nonstandard management of sterile articles in clinical departments has reached 18.21%, mainly in the four links of receiving, distribution, storage, and use [11, 12]. The management of sterile articles in clinical departments ensures patient safety. The quality control of the final use of sterile articles in departments has attracted more and more attention from nursing experts [13–15]. Clinical nurses lack understanding of the standardized management of sterilized articles [16]. Therefore, the staff of the disinfection supply center should give full play to their professional ability and improve the standardization of the management of sterilized articles in clinical departments with a scientific and standardized attitude under the guidance of the nursing department and infection control department. It can be seen from Table 5 that the qualified rate of sterile articles management after the clinical department was assisted by the disinfection, and supply center has been dramatically improved compared with that before the rectification. After the nursing department incorporated the standardized management of clinical, sterile articles into the quality control inspection of the nursing department, the disinfection and supply center found that the nurses in the clinical department had a great improvement in the management awareness of sterile articles. The head nurse has also strengthened the supervision of sterile goods management. After the head nurse of the disinfection supply center gave standardized online and offline teaching and training on the management of sterile items, it was found that the nonstandard problems of counting records and storage environment of sterile articles in clinical departments had decreased significantly, reducing the loss of sterile bags caused by nonstandard management and reducing the workload of staff in the disinfection supply center and the loss of hospital costs. At the same time, during the inspection, we also found that the work of the disinfection supply center was not done in place. For example, the packaging found in the inspection was not standardized. After the inspection and analysis, some workers grabbed the sterile package hard when distributing the sterile package, resulting in the loose packaging of the sterile package, which was corrected later to improve the work quality of the disinfection supply center. From Table 1, Table 3, and Table 4, it was found that the problem that the sterile package is not normally placed according to the expiration date has always been the main problem in the problem composition ratio, and the improvement is not obvious. We found that the user is not familiar with the equipment in the package when taking the sterile package, and the problem occurs from time to time when he puts it back into the bacteria-free cabinet after taking the wrong one. Therefore, how to improve the awareness of clinical users of sterile devices in the package is what we need to study in the future. At the same time, it was also found that the proportion of damaged sterile bags increased from none to 21.4%, which became the main problem after rectification. After the inspection and understanding by the disinfection supply center, it was found that with the strengthening of the management of sterile articles by clinical departments, the frequency of checking sterile articles every day was increased. It resulted in minimal damage after the wear of paper and plastic packaging, which was challenging to find.

The article "The Supervision and Management Mode of Disinfection Supply Center Improves the Standardization of Sterile Goods Management in Clinical Departments" was retracted in 2023. Reasons: unreliable results or conclusions; concerns about the data; concerns about the results or conclusions; concerns about the peer review.

The disinfection supply center is an important service department of clinical departments [17]. While doing an excellent job cleaning, disinfection, and sterilization, we should give full play to our professionalism and actively do an extended service of clinical departments. The specialty can best reflect their life value [18]. As the staff of the disinfection supply center, they can give full play to their professional ability in managing sterile articles, actively participate in and assist the management of sterile articles in clinical departments, and promote the effective implementation of this work to a great extent. More and more researchers [19, 20] in China pay attention to standardizing the management of the sterility effectiveness of sterile articles before use. They have also carried out research and improvement in various aspects. This paper also summarizes and improves various studies and puts forward the supervision mode of disinfection supply center. The specific content is to formulate and improve relevant management systems for the storage and use of sterile clinical articles in the hospital under the guidance and assistance of the hospital nursing department and the hospital feeling department, led by the disinfection supply center and according to the sterile article management specifications of the disinfection supply center. In addition, the staff of the disinfection supply center shall inspect the standardized management of sterile articles in relevant departments of the hospital once a quarter, supervise and correct the problems, summarize them at the same time, and include them into the careful management of sterile articles in the quality control inspection of the nursing department for scoring. The disinfection supply center shall summarize and analyze the inspection results in that year and analyze and improve the existing main problems.

The article "The Supervision and Management Mode of Disinfection Supply Center Improves the Standardization of Sterile Goods Management in Clinical Departments" was retracted in 2023. Reasons: unreliable results or conclusions; concerns about the data; concerns about the results or conclusions; concerns about the peer review.

To sum up, the nursing department will incorporate the standardized management of the storage and use of sterile articles in clinical departments into the nursing quality inspection. By adopting the supervision and management mode of disinfection supply center, the disinfection supply center will regularly supervise the sterile articles in clinical departments, provide targeted training and on-site guidance to rectify existing problems, and strengthen the critical concept of standardized management of sterile articles by clinical medical staff. It ensures the closed-loop management of sterilization effectiveness of sterile articles and safe use which improve the standardized management and safe use of sterile articles in clinical departments. At the same time, it can also reduce the cost consumption caused by the loss of sterile packages.

## Figures and Tables

**Table 1:** Problems of sterile articles inspected in clinical departments from April to June 2018.

Existing problems	Total inspection frequency	Frequency of problems	Composition ratio (%)
Aseptic bags are not properly placed according to the expiration date	65	9	16.7
	65	6	11.1
The storage environment does not meet the requirements	65	2	3.7
	65	3	5.5
There are expired packages not taken out	65	26	48.1
	65	7	13.0
The label of sterile bag is damaged	65	1	1.9
	65	0	0
The base number of sterile packages is inconsistent with the record	520	54	100

**Table 2:** The clinical department personnel participated in the training record of sterile material management.

Training period	Training method	Number of training departments	The number of participants
Rectification	On-site intensive training	65	138
Rectification	Online medical classroom training	65	1265
Rectification	Department self-training	65	982

The article "The Supervision and Management Mode of Disinfection Supply Center Improves the Standardization of Sterile Goods Management in Clinical Departments" was retracted in 2023. Reasons: unreliable results or conclusions; concerns about the data; concerns about the results or conclusions; concerns about the peer review.

**Table 3:** Problems of sterile articles in clinical departments from July 2018 to June 2019.

Existing problems	Total inspection frequency	Frequency of problems	Composition ratio (%)
Aseptic bags are not properly placed according to the expiration date	260	13	32.5
	260	13	32.5
The storage environment does not meet the requirements	260	6	15
	260	2	5
There are expired packages not taken out	260	0	0
	260	0	0
The label of sterile bag is damaged	260	2	5
	260	4	10
In total	2080	40	100

**Table 4:** Problems of sterile articles in clinical departments from July 2019 to June 2021.

Existing problems	Total inspection frequency	Frequency of problems	Composition ratio (%)
Aseptic bags are not properly placed according to the expiration date	520	13	46.4
	520	3	10.7
The storage environment does not meet the requirements	520	4	14.3
	520	1	3.6
There are expired packages not taken out	520	0	0
	520	0	0
The label of sterile bag is damaged	520	1	3.6
	520	6	21.4
In total	4160	28	100

**Table 5:** Comparison of qualified rates of sterile articles in clinical departments.

	Existing problems	Total inspection frequency	Frequency of problems	Composition ratio (%)
Before rectification	520	54	466	89.5
Rectification in progress	2080	40	2040	97.5
After rectification	4160	28	4132	99.4
*χ* ^2^	67.988			
*P*	<0.001			

**Table 6:** Comparison of number and value of lost packages in clinical departments (*n* = 325).

	Average number of lost packages (rate)	Loss value (yuan)
Before	34(10.5%)	1190
In progress	7(2.2%)	230
After	2(0.6%)	70
*χ* ^2^	43.257	
*P*	<0.001	

## Data Availability

The data used to support the findings of this study are included within the article.
